The article "The long-term effect of body contouring procedures on the quality of life in morbidly obese patients after bariatric surgery" was published in 2020. Journal: PLoS One.

# The long-term effect of body contouring procedures on the quality of life in morbidly obese patients after bariatric surgery

**DOI:** 10.1371/journal.pone.0229138

**Published:** 2020-02-21

**Authors:** Marek A. Paul, Jakub Opyrchał, Michał Knakiewicz, Paweł Jaremków, Łukasz Duda-Barcik, Ahmed M. S. Ibrahim, Samuel J. Lin

**Affiliations:** 1 Department of Plastic Surgery, DSS, im. T. Marciniaka, Wroclaw, Poland; 2 Division of Plastic and Reconstructive Surgery, Beth Israel Deaconess Medical Center, Harvard Medical School, Boston, Massachusetts, United States of America; Universitatea de Medicina si Farmacie Carol Davila Biblioteca, ROMANIA

## Abstract

**Introduction:**

There has been a significant increase in the number of body contouring procedures performed worldwide. This study aimed to evaluate the long-term psychosocial effects of these procedures among patients who undergone weight loss surgery and maintained their body mass for a minimum of one year.

**Material and methods:**

Post-bariatric patients undergoing body contouring procedures were recruited for the study consecutively. Inclusion criteria: BMI < 30 following bariatric surgery, weight maintenance for a minimum of 12 months, and completion of all follow up questionnaires (6 and 12 months). Patients were surveyed 24 hours before, 6-months, and 12-months post-procedure using a Polish validated version of BODY-Q.

**Results:**

30 consecutive patients with a mean age of 38 years (SD 5,91) were included in this study. The BODY-Q questionnaire revealed statistically significant improvements in the acceptance of body appearance after 12 months of follow up. In the abdominal area, the rise in scores achieved 90 from the starting level of 13, and the overall body image increased from 24 to 67. Moreover, in patients with postoperative complications (one hematoma and four minor wound dehiscence), the overall score did not differ from uncomplicated patients.

**Conclusions:**

Body contouring procedures after massive weight loss significantly improve the general perception of personal appearance as well as both the psychological and social aspects of life in patients, already significantly stigmatized by their appearance. Body contouring procedures have essential value and should be widely offered as a step in the treatment of morbidly obese patients.

## Introduction

Obesity and being overweight contribute to more deaths in a majority of the World’s population than undernourishment. [1] As a result, interest in bariatric surgery within this patient population has risen. However, this method of treatment exhibits various consequences, among which the skin excess and loss of its elasticity are the most common. Up to 89% of post-bariatric patients develop sagging of the skin most prominent in the upper arms and abdominal area. [2] It does not only affect self-perception, but it also influences psychological, social, and sexual well-being. [3] According to the latest available ISAPS global statistics, body and extremities procedures increased by 7% within just one year, reaching the total number of almost three and a half million surgeries performed annually.

What is more, in 2017, the lower body lift showed the second largest, after vaginal rejuvenation, an increase in a number of procedures with a 22% rise. [4] It is an excellent example of how body contouring procedures continue to gain popularity. In Poland, surgical removal of skin excess in patients after massive weight loss, with appropriate qualification, is covered by the National Healthcare Insurer. Body contouring procedures aim to help overweight and obese patients to regain self-confidence.

Thus far, we have limited data on the long-term psychosocial outcomes in patients who have undergone massive weight loss, followed by a body contouring procedure. Klassen et al. noted a shortage of evidence on meaningful patient outcomes within the literature for this patient population, in particular, health-related quality of life (HRQoL), body image, and satisfaction with appearance. To evaluate relevant results a highly specific patient-reported outcomes instrument is required. As such, we utilized a previously developed official Polish translation of the BODY-Q questionnaire—a Patient—Reported Outcome (PRO) Instrument for Weight Loss and Body Contouring (BC) treatments. [5–7] Our study aimed to evaluate the long-term psychosocial outcomes of body contouring procedures using the BODY-Q questionnaire, by comparing pre- and post- BC results with 12 months of follow up, among post-bariatric patients recruited consecutively over 2-year-period.

## Materials and methods

### Patient population and enrollment

A prospective, single-institution study was conducted among 30 consecutive patients that underwent a body-contouring procedure between 2015 and 2017. Inclusion criteria comprised patients older than 18 years old, with BMI less than 30, and having a stable weight for 12 months following bariatric surgery who presented skin sagging and redundancy resulting in clinical manifestations such as chronic skin infections, prolonged skin rashes, ulcerations, and functional limitations. Data regarding demographics and medical history were collected from patient records. All patients received at least a minimum of a 12-month follow-up postoperatively. The study was granted an exemption in writing by the Lower Silesian Hospital Board of Quality Control and Study IRB Department, represented by the Chief of the Medical Section of the Hospital. This study followed the Declaration of Helsinki on medical protocol and ethics. All patients signed the informed consent about the study at the time of enrollment before any study procedures were done. All data were deidentified after study end, and all patients completed the study.

### Clinical outcomes assessment

For the study, an official Polish translation and language validation of the Body-Q was done in adherence to the Translation and Cultural Adaptation group (TCA group) principles and World Health Organization (WHO) guidelines on translation and adaptation of instruments. [8, 9] Twenty-four hours before surgical intervention, all participants completed the validated Polish version of BODY-Q questionnaire. The structure of the BODY-Q survey used in this study adheres to the recommended methods for the development of a patient-reported outcomes instrument. [10, 11] The goal of the questionnaire was to ascertain patients’ perceptions of weight loss and body contouring based on three metrics: health-related quality of life, physical appearance, and the process of care.

The preoperative surveys were conducted in a pen-and-paper format. In the postoperative period, the survey was sent to patients via a secured email. Patients were contacted by phone a week before emails were sent out and informed to check their inbox. If no information was received within two weeks, patients were contacted and reminded with another phone call. The preoperative survey contained an additional title page with demographic information, type of bariatric surgery as well as weight before and after massive weight loss (Table 1). The preoperative module consisted of 14 metrics: appearance scales (body, abdomen, buttocks, back, outer thighs/hips, inner thighs, upper arms, skin excess) and HRQoL scales (body image, psychological function, social function, sexual well-being, physical function, physical symptoms related to obesity). Although the last two subscales are specific to patients with obesity, we used them to assess the persistence of any symptoms in post-bariatric patients. The postoperative module included an additional four scales inquiring about patients’ experiences related to treatment, and appraisal of body contouring scars. When the postoperative module was being filled out, patients were not permitted to reference their preoperative answers.

**Table 1:** Patient demographics.

Characteristics	Number of patients n = 30 (%)
Age: Mean ± SD, years	38 ± 5,91
BMI before massive weight loss	
Class II obesity (35,0–39,9 kg/m2)	2 (7%)
Class III obesity (>40,0 kg/m2)	28 (93%)
BMI after massive weight loss	
Normal (18,5–24,9 kg/m2)	12 (40%)
Overweight (25,0–29,9 kg/m2)	12 (40%)
Class I obesity (30,0–34,9 kg/m2)	6 (20%)
Education	
Elementary	1 (3%)
High School	21 (70%)
Graduate	8 (27%)
Marital status	
Single	9 (30%)
Married	15 (50%)
Divorced	6 (20%)
Employment status	
Employed	17 (57%)
Unemployed	13 (43%)

### Body contouring procedures

Three plastic surgeons from our department performed all surgeries. Patients underwent various body contouring procedures, depending on the preoperative assessment and the best—predicted outcome for the patient. Our patient population was subject to a vast array of body contouring procedures depending on the surgical indication. Procedures were performed in a standard fashion using high lateral tension abdominoplasties without liposuction, and quilting sutures used. [12] Each of our patients was asked to use compression garments for four weeks after surgery. Some of our patients had a lower body lift procedure performed. The operation was executed in a standard fashion as described by Aly et al.; a 360-degree incision was used to resect excess tissue in the abdominal, thigh, and buttock areas. [13] No liposuction was performed in these patients. Additional contouring operations included thigh lift and brachioplasty. Thigh lifts were performed using a full T incision as described by Hurwitz with additional liposuction or only inguinal resection with liposuction. [14] Brachioplasty was performed according to Hurwitz et al.; utilizing liposuction and an L shaped skin incision in all patients. [15]

All patients had preoperative compression garment thromboembolism prophylaxis, and low molecular weight heparin (LMWH) administered following hospital protocols. We used the Caprini Risk Score to stratify our patients for venous thromboembolism risk. LMWH was given to all the patients with Caprini score at least 3 or higher. [16] Depending on the patient’s risk group, we administered the first dose 12 hours before surgery, and it was continued daily for 7–14 days. Due to higher probability of DVT rate in abdominal and lower-body lift procedures the LMWL prophylaxis was given 14 days in comparison to 7 days in other body contouring procedures. All patients were mobilized the same day after the procedure to lower their risk of a possible thromboembolic incident.

### Statistical analysis

Data were compared using the t-test. The raw scores from the tables were converted into a scale ranging from 0 to 100 by the Rasch model. [17] Data analyses were performed using IBM SPSS Statistics, version 24.0 (Armonk, NY: IBM Corp.) A value of p <0,05 was considered statistically significant.

## Results

### Patient characteristics

A total of 30 patients met our inclusion criteria and were enrolled in the study. The overall survey response rate was 86%. All male patients (n = 2) refused to fill out the BODY-Q questionnaire and were excluded from the analysis. As such, the final study group consisted of female patients only. Patients undergoing BC were, on average, 38 years old (SD 5.91) with an average weight loss of 53.1 kg (SD 5.02). Detailed characteristics of our patient population are presented in Table 1.

### Procedures performed

Participants have undergone laparoscopic sleeve gastrectomy (LSG), adjustable gastric banding (AGB), and Roux-en-Y gastric bypass (RYGB) with the mean period of 34 months from body contouring (Table 2). A total of 41 BC procedures were performed in 30 patients (Table 3). The most common body contouring procedure was abdominoplasty (n = 22; 54%) followed by lower-body lift (n = 7; 17%). The three fourth of patients (n = 22; 73%) underwent a single BC procedure. The remaining eight had anywhere from 2 to 4 surgeries performed. The mean operative time (MOT) for lower body lift was 217.5 minutes, and length of hospital stay (LOS) was five days followed by abdominoplasty patients with MOT of 133.9 minutes and LOS of 4.9 days. Complications occurred in five patients (16.7%), one hematoma (3.3%), and wound dehiscence in four patients (13.3%). As hematoma required wound revision in the OR in the third postoperative day, it was classified as a major complication. Nevertheless, the patient did not demand blood transfusion. All other patients with wound dehiscence were classified as minor complications, treated conservatively with dressing change.

**Table 2:** Procedures performed for body contouring in post-bariatric patients.

Bariatric Procedure	Number of patients (%)
Laparoscopic sleeve gastrectomy (LSG)	20 (67%)
Adjustable gastric banding (AGB)	6 (20%)
Roux-en-Y gastric bypass (RYGB)	4 (13%)

**Table 3:** Distribution of bariatric procedures for patients undergoing body contouring surgery.

Body Contouring Procedure	Number of procedures (%)
Abdominoplasty	22 (54%)
Lower body lift 360	7 (17%)
Inner thighs	6 (15%)
Outer thighs	2 (5%)
Upper arms	2 (5%)
Buttocks	1 (2%)
Back	1 (2%)
Total	41 (100%)

### Outcomes of the Body-Q questionnaire

The maximum number of points on each scale is 100. Higher scores correlate with greater satisfaction. There were statistically significant improvements observed in the acceptance and evaluation of body appearance in the postoperative module (p<0,001) (Fig 1). The worst satisfaction at baseline was observed in the abdominal and thigh region.

**Fig 1:** Comparison of satisfaction with appearance of different body regions before and after body contouring surgery.

Moreover, health-related quality of life was significantly enhanced (≥ 20 points) with regards to psychological well-being, social functioning, sexual well-being, and body image (p<0,001) (Fig 2). Furthermore, in 15 (50%) of the studied patients, surgery in at least one region positively affected the perception of the rest of the body. In three patients (10%), we noted a decreased satisfaction with untreated body areas. Our analysis did not show any significant difference in the final satisfaction rate between patients who underwent only one BC procedure and those who had multiple procedures performed (71.36±17.15 vs. 73.38±19.02; p = 0,79).

**Fig 2:** Comparison of satisfaction with quality of life before and after body contouring surgery.

## Discussion

The emergence of body contouring procedures has paralleled the rising trend in bariatric surgery for massive weight loss. [18, 19] Patients seek a solution for redundant, unattractive, and loose skin, refractory to diet and physical exercise to achieve what is deemed a “natural look.” Studies have shown that this, in turn, improves functional and aesthetic results and reduces psychological burden. [20–22] These procedures have the potential to restore proper form and tissue structure. [23, 24]

We believe that our high response rate (86%), despite the time-consuming survey, is associated with collecting the questionnaires in pen-and-paper form. On the other hand, it is hard to analyze hand-written data in bigger study groups, so it is more convenient and accurate to obtain electronic data capture for further studies. Also, as reported by Geerards et al., reduced assessment length using BODY-Q computerized adaptive testing could reduce patient burden while preserving the accuracy of clinical patient-reported outcomes. [25]

In our study, average weight loss was 53.1 kg. Weight loss was achieved following a bariatric operation as previously described, and after that weight remained stable for at least 12 months. It is contrary to reports by Balagué et al., and Felsenreich et al., that 5 percent of patients regain weight a year after surgery; this was not observed in our cohort. [26–28] The mean age of patients in our study was 38 years old, which is younger than in previously published studies. [29–31] Perhaps, this can be attributed to the ease of access to care and increased knowledge about weight loss options in Poland. The significance of patients supports groups that share information about post-bariatric treatment might also be an essential factor. Although the first procedures performed in Poland were described in the 1970s, an early survey defining the current status of bariatric operations was popularized in 2007, and a substantial rise in the number of surgeries performed was observed in 2014. [32, 33] A majority of study participants underwent abdominoplasty followed by the lower body lift. It is consistent with previously reported problematic parts of the body following massive weight loss surgery. Mitchell et al., found abdominoplasty to be the most commonly performed procedure following bariatric surgery, accounting for 24.3 percent. [23] This notion is echoed by Giordano et al., who observed that the waist/abdominal region was operated on in 62.2 percent of post-bariatric patients. [24]

Our study objectively assesses whether body contouring procedures positively impacted the lives of patients after bariatric surgery. It was achieved using the BODY-Q survey. Interestingly the lowest preoperative (13 points) and highest postoperative (90 points) scores for appearance satisfaction were observed for abdominoplasty. It is reinforced in a study by Poulsen et al. [34] Moreover, there was a statistically significant improvement in body perception across all operated body regions postoperatively. However, it is essential to note that the quality of life in the postoperative period was not linked to the number of regions operated. None of the surveyed patients was dissatisfied with the outcome of the procedure. Health-related quality of life was significantly enhanced in all operated-on body areas across all life scales, with the highest change noted in the body image. Song et al. noted a similar observation despite the use of a different, less coherent, assessment scale—the Body Image and Satisfaction Assessment scale (BISA) on a smaller patients’ sample. Although, we did not observe that surgical modification of one area led to dissatisfaction in other parts of body, rather we noted opposite reaction when patient was more satisfied with the rest of the body. However, based on clinical experience may suggest that as proposed by Song et al. correction of one body part my lead to exposure of other parts and consequently result in dissatisfaction. [29] As we noted in the results, the surgery in at least one region positively affected the perception of the rest of the body.

In our group, the complication rate was found to be 16.7%. We did not observe any correlation between lower satisfaction rates in patients with those minor or even major complications. This is comparable to complication rates reported by Winocour et al., and Chong et al., and lower than that in a study done by Au et al. [35, 36] The mean hospital stay in our group was around five days, which is longer than presented in other studies, which is contributed by a more extended pre- and postoperative stay, mainly due to the reimbursement requirements set by the National Health Fund regarding the LOS. [37] The main discharge criterion was the drain removal, with fluid output less than 30-40cc. Our choice of BODY-Q survey was preceded by a long data base search. Currently, BODY- Q seems the most universal questionnaire that may be applied to patients worldwide after careful and validated translation. In 2014, Klassen et al compared BODY-Q to other HR-QOL surveys such as Moorehead-Ardelt Quality of Life Instrument (MAQOL), Quality of Life–Lite (IWQOL-Lite) instrument or Swedish Obese Subjects Obesity. [6] The major benefit of BODY-Q is that it allows to measure not only HR-QOL but also appearance-related concerns and the patient experience of health care. The versatility and precision of this instrument was reported later by Poulsen et al. who compared BODY‐Q with Moorehead‐Ardelt quality of life questionnaire‐II (MAQOL‐II) proving MAQOL‐II hat does not meet today’s standards for a rigorously developed PRO measure. [38]

The strength of this study was using a worldwide approved validated questionnaire, long—term follow up (up to 12 months), and a high response rate of 86%. In contrast to previously published BODY-Q questionnaire-related studies, which are cross-sectional and lack longitudinal assessment, the survey was administered to our patient population 24 hours before, six, and twelve months after their body contouring procedure. [34, 39]

The limitation of this study was a relatively small number of surveyed patients (30), only females, the possible impact of “no pay” procedure as paid by the National Health Insurance.

Moreover, this study showed the highest satisfaction rate for abdominoplasty patients. It could be biased as the abdominoplasty had the highest number of procedures done among the small group, and other surgeries may not achieve enough statistical power. We plan to focus our subsequent studies on the least reported body contouring surgeries to gain more knowledge about those specific procedures. For future studies, we plan on using a more efficient means of data acquisition such as EDC software (IBM Watson Health), rather than “pen and paper” approach or manually emailed surveys. It will better ensure data safety and minimize human error.

## Conclusions

As the study presents, Poland does not differ from other countries in the growing demand for bariatric and post-bariatric procedures. We proved the significant impact of improved body assessment after body contouring procedures. We still need more data on the specific characteristics of patients that profoundly change their perception of their surgical outcomes.

We have shown that these procedures lead to a significant improvement in both the psychological and social aspects of patients’ lives. Finally, the BODY-Q is an easy and efficient tool that may provide greater insight for result optimization within this patient population.

## Supporting information

S1 File (XLSX)
